The article "The Role of Posttranslational Modification and Mitochondrial Quality Control in Cardiovascular Diseases" was retracted in 2023. Reasons: signs of a paper mill; suspected computer-generated content; unreliable results or conclusions; concerns about the data.

# The Role of Posttranslational Modification and Mitochondrial Quality Control in Cardiovascular Diseases

**DOI:** 10.1155/2021/6635836

**Published:** 2021-02-18

**Authors:** Jinlin Liu, Li Zhong, Rui Guo

**Affiliations:** ^1^College of Life Sciences, Institute of Life Science and Green Development, Hebei University, Baoding 071002, China; ^2^College of Osteopathic Medicine of the Pacific, Western University of Health Sciences, Pomona, California, USA

## Abstract

Cardiovascular disease (CVD) is the leading cause of death in the world. The mechanism behind CVDs has been studied for decades; however, the pathogenesis is still controversial. Mitochondrial homeostasis plays an essential role in maintaining the normal function of the cardiovascular system. The alterations of any protein function in mitochondria may induce abnormal mitochondrial quality control and unexpected mitochondrial dysfunction, leading to CVDs. Posttranslational modifications (PTMs) affect protein function by reversibly changing their conformation. This review summarizes how common and novel PTMs influence the development of CVDs by regulating mitochondrial quality control. It provides not only ideas for future research on the mechanism of some types of CVDs but also ideas for CVD treatments with therapeutic potential.

## 1. Introduction

Cardiovascular disease (CVD) is currently one of the most perplexing diseases because of its variety and complexity. The mortality rate of CVDs, accounting for 30% of the death toll in the world, has still been increasing every year [1, 2]. CVDs not only affect human life but also cause great socioeconomic burden. Thus, coronary artery disease is considered one of the major CVDs affecting the global human population and has been considered as a major cause of death in both developed and developing countries [3]. Coronary artery disease can cause severe myocardial infarction and contributes to the development of heart failure [4]. However, the pathologic process and risk factors of CVDs are still controversial, especially the molecular mechanisms on modulating mitochondria-associated proteins by posttranslational modifications (PTMs) [5, 6].

The mitochondrion, a membrane-bound organelle, is present in all eukaryotic cells. It is crucial to maintain the normal mitochondrial function to provide energy for cell survival. Therefore, disturbed mitochondrial quality control and homeostasis can result in a variety of CVDs. Mitochondrial biogenesis, fusion, fission, mitophagy, and protein turnover are considered as the main processes for mitochondrial quality control [7–12]. Dysfunctional mitochondria or mitochondrial proteins are degraded and removed by the ubiquitin-proteasome system (UPS) or by autophagy (mitophagy) to maintain a normal mitochondrial homeostasis [13, 14]. PTMs refer to the chemical modifications of specific amino acid residues of proteins, the reactions of which are mostly reversible [15]. A majority of the proteins in cells undergo PTMs by changing their structures and functions by conformational alterations [16]. PTMs of proteins have been shown to affect mitochondrial quality control, thereby exacerbating or alleviating CVDs [17–19]. Therefore, the purpose of this review is to summarize the functional changes of intracellular proteins especially mitochondrial-related proteins by PTMs and their effects on CVDs, particularly myocardial ischemia/reperfusion (I/R) injury, myocardial infarction, and heart failure. The PTMs including acetylation, phosphorylation, SUMOylation, ubiquitination, succinylation, lactylation, and crotonylation are discussed, and they shed light on a theoretical basis of CVD treatment in the future.

## 2. Mitochondrial Quality Control and Cardiovascular Diseases

Mitochondria are cellular organelles involved in energy production in the form of ATP through the process of oxidative phosphorylation, citric cycle, and *β*-oxidation to maintain cardiomyocyte vitality [20]. The mitochondrial environment has thus emerged as a key part in the pathogenesis and progression of CVDs which eventually can lead to heart failure. Mitochondrial fission and fusion, as well as mitophagy, are major processes in maintaining mitochondrial quality control, of which fission and fusion are primarily mediated by the following three particular proteins: (1) optic atrophy 1 (OPA1), localized to the inner membrane of mitochondria (IMM), which can move to the intermembrane space (IMS) and play a unique role in IMM fusion to crest structure adjustment; (2) mitofusins 1 and 2 (Mfn1 and Mfn2), which are located in the outer membrane of mitochondria (OMM) for OMM fusion [21]; and (3) dynamic protein-related protein 1 (Drp1), which is generally located in the cytoplasm and can be transferred to the mitochondria to divide the OMM and mediate the process of mitochondrial fission. Similarly, there are multiple ways to remove damaged mitochondria, such as degradation by proteasomes, combination with mitophagy, and fusion with a lysosome. In a word, the abnormality in mitochondrial quality control that is regulated by a complex network will cause severe mitochondrial disturbance.

There are plenty of mitochondria in cardiac cells for the high energy demand of the heart. ATP synthesis and energy metabolism cannot be performed normally in patients with mitochondrial defects [22]. On the other hand, mitochondrial dysfunction can cause a variety of CVDs or cardiac disorders such as cardiac I/R injury, myocardial infarction, cardiac hypertrophy, and heart failure [23, 24]. Damaged mitochondria are not able to synthesize sufficient ATP, but they increase the reactive oxygen species (ROS) levels. ROS is a major by-product during the process of mitochondrial respiration. Excessive cellular ROS contents not only cause loss of certain DNAs and proteins but also lead to the occurrence of heart failure and other diseases [25–28]. To this end, understanding the mechanisms of mitochondrial quality control and the degradation of unhealthy mitochondria or abnormal mitochondrial proteins plays an important role in maintaining normal cardiac function.

## 3. The Main Types of Mitochondrial PTMs in Cardiovascular Disease

### 3.1. SUMOylation

Small ubiquitin-like modifiers (SUMO), with a molecular weight of about 10 kDa, belong to the large family of ubiquitin-like (Ubl) proteins. There are four subtypes of SUMO in mammals, namely, SUMO1, SUMO2, SUMO3, and SUMO4 [29–32], of which SUMO2 and SUMO3 have about 97% similarity [33]. The subtypes SUMO1-SUMO3 are widely expressed, while SUMO4 is only expressed in the kidney, spleen, and lymph nodes [34–36]. SUMOylation is classified as a ubiquitination-like PTM, binding the SUMO protein to the lysine residue of the substrate protein through successive steps of reactions by the SUMO activating enzyme (E1, a heterodimer of SAE1/SAE2 subunits), the SUMO conjugating enzyme (E2, also known as Ubc9), and several E3 ligases with ATP consumption (see Figure 1) [37]. At present, only one type of E1 or E2 has been found whereas there are more than ten types of E3 ligases, which are divided into three categories: protein inhibitor of activated STAT (PIAS) proteins, Ras-related nuclear protein binding protein 2 (RanBP2), and human polycomb 2 (Pc2)/Chromobox 4 (CBX4) [38, 39]. The SUMOylation process is reversible. Importantly, SUMO-specific proteases such as cysteine proteases of the sentrin-specific protease (SENP) family (including SENP1-SENP3 and SENP5-SENP7) are involved not only in the activation of SUMO precursors but also in the separation of SUMO and substrate proteins [33, 37]. Evidence has shown that SUMOylation is involved in mitochondrial quality control, cytochrome C release, and Ca^2+^ homeostasis of cardiomyocytes [40, 41]. As a result, in recent years, more and more attention has been paid to the role of mitochondrial protein SUMOylation in CVDs.

#### 3.1.1. Mitochondrion-Related Protein SUMOylation in Myocardial I/R Injury

Drp1, a GTPase, is not only associated with mitochondrial fission but is also involved in mitochondrial apoptosis [42]. The SUMOylation modification of Drp1 has a great impact on mitochondrial quality control and plays a crucial role in cardiac I/R injury. Previous research indicated that following I/R injury of the heart, the binding capacity of SUMO1 to Drp1 increased and formed a complex. Zinc promoted mitochondrial fission by increasing the acidification of the complex, thereby eliminating damaged mitochondria and maintaining mitochondrial quality stability, further improving cardiac function [43]. Evidence revealed that SENP3, an enzyme of deSUMOylation, was associated with apoptosis induction in response to cardiac I/R by affecting Drp1 localization in the mitochondria. However, mdivi-1, an inhibitor of Drp1, alleviated myocardial damage by inhibiting the expression of SENP3 [44].

#### 3.1.2. Mitochondrion-Related Protein SUMOylation in Heart Failure

In both mouse models and humans, a low level of apoptosis in cardiomyocytes is detrimental to the heart and may contribute to the progression of heart failure [45, 46]. Kim et al. found that SENP5 expression was significantly higher than normal in heart failure [47]. Drp1, a pivotal protein that mediates the apoptosis of cardiomyocytes, was induced by SENP5 which has long been shown to be of great significance for regulating mitochondrial function [48]. Data revealed that SENP5 activity was reduced by apoptotic factors after deletion of Drp1 in cardiomyocytes. On the contrary, upregulation of SENP5 expression elevated mitochondrial apoptosis levels via the connection between Drp1 and SUMO2/3 [47].

### 3.2. Ubiquitination

The ubiquitin-proteasome system (UPS) is the primary system of protein degradation in eukaryotic cells. Ubiquitin is a polypeptide containing 76 amino acids, and ubiquitination occurs by covalently binding its own COOH group at the glycine end with the free *ε*-NH2 terminus of a lysine residue in the target protein [49, 50]. Each ubiquitin has multiple binding sites for the combination with other ubiquitin peptides to form ubiquitin chains. The binding of the ubiquitin molecule to the lysine residue of the target protein will initiate the degradation of marked proteins [51]. In addition to binding to lysine residues, ubiquitin can also combine with the amino terminus of the substrate [52]. Ubiquitination is a cascade reaction coordinated and catalyzed by E1 (ubiquitin activating enzyme), E2 (ubiquitin conjugating enzyme), and E3 (ubiquitin ligase), and the process is also reversible (see Figure 2) [49, 53]. Similar to SENPs, deubiquitinases (DUBs) are capable of activating ubiquitin precursors by splicing or removing ubiquitin molecules from tagged proteins [54]. Ubiquitination has been widely studied as protein degradation is the major way to maintain mitochondrial quality and intracellular homeostasis.

#### 3.2.1. Mitochondrion-Related Protein Ubiquitination in Myocardial I/R Injury

There are varieties of ubiquitin E3 ligases reported in human cells, which are vital for the ubiquitination process. Parkin, an E3 ligase, can ubiquitinate several mitochondrial outer membrane proteins through its E3 ligase activity to recruit the p62 protein, which interacts with LC3, leading to the process of PINK/Parkin-mediated mitophagy [55]. Evidence has shown that expression of Parkin is beneficial to cardiac function, specifically, by catalyzing CypD ubiquitination in the cell necrosis cascade and inhibiting the opening of the mitochondrial permeability transition pore (mPTP), therefore alleviating myocardial injury [56]. Another study found that Tongxinluo, a medicine for treating coronary heart disease, was involved in activating Parkin and reducing the activity of the ubiquitin system to attenuate myocardial I/R injury [57], although few studies have reported which particular or active ingredients of the Tongxinluo capsule may play a regulatory role in the PINK/Parkin pathway [58, 59]. Phosphatase and tensin homolog (PTEN) is a tumor-suppressor protein located in mitochondria [60]. Li et al. revealed that the terminal end of PTEN can bind to the E3 ligase Parkin and promote the translocation of Parkin within mitochondria. The loss of PTEN was reported to be more susceptible to the I/R injury of the heart, due to its ability to induce structural and functional abnormalities of the mitochondria in mouse cardiomyocytes [54]. In the process of heart remodeling following I/R injury, exogenous ubiquitin treatment significantly reduced Caspase-9 expression in the mitochondrial death pathway, reduced infarct area, increased mitochondrial production, and finally improved heart function. In short, ubiquitination is closely associated with myocardial I/R injury [61].

#### 3.2.2. Mitochondrion-Related Protein Ubiquitination in Cardiomyopathy

Mutations in E3 ligases MuRF1 and MuRF2 are critical for the development of hypertrophic cardiomyopathy (HCM). In patients with HCM, increased MuRF1 mutants in adult cardiomyocytes resulted in a reduction of ubiquitination, as well as UPS-mediated degradation of myosin heavy chain 6 (Myh6) and cardiac myosin-binding protein-C (cMyBP-C) [62]. Parkin is necessary for mitochondrial quality control, and its expression is relatively low in a normal heart. It was suggested that the ablation of Drp1 inhibited mitochondrial fission by promoting Parkin expression, which in turn led to cardiomyopathy [63]. In addition, another study found that disturbed mitochondrial redox status induced by lipid toxicity eventually led to mitochondrial dysfunction and cardiomyopathy, the mechanism of which may be due to an enhanced mitochondrial fission through increased AKAP121 (A kinase anchor protein 121) ubiquitination that resulted in a reduction in Drp1 phosphorylation at the site of Ser637, as well as the changes in OPA1 protease hydrolysis [64].

#### 3.2.3. Mitochondrion-Related Protein Ubiquitination in Heart Failure

Both coronary artery disease and cardiomyopathy contribute to the development of heart failure. One of the reasons that trigger heart failure is the excessive death of cardiomyocytes. For instance, a certain extent of mitophagy is accompanied with the clearance of damaged mitochondria, the improvement of mitochondrial function, the reduction in ROS production, and the apoptosis of cardiomyocytes. However, excessive mitophagy can cause cardiac injury because of cell death. Evidence has shown that PINK1-associated ubiquitination and phosphorylation enhanced mitochondrial depolarizing by raising Parkin activation and recruitment, causing increased mitophagy via the PINK1-Parkin-SQstm1 (Sequencesome-1) pathway. In addition, alanine mutation of PINK1 at Ser495 partially inhibited AMPK*α*2 overexpression-induced mitophagy and improved the mitochondrial function stimulated by phenylephrine in cardiomyocytes. In failing hearts, however, the dominant AMPK*α* isoform switched from AMPK*α*2 to AMPK*α*1, exacerbating the heart failure condition [65]. Moreover, the results obtained by Yang et al. indicated that leptin enhanced OPA1 by inhibiting the activity of OMA1, a mitochondrial protease. In this process, GSK3 phosphorylation was a prerequisite for ubiquitination-dependent degradation of OMA1, thereby attenuating OPA1 cleavage. Additionally, leptin induced mitochondrial fusion and improved mitochondrial respiratory function in hypoxic hMSCs (human mesenchymal stem cells), indicating a protective role of leptin against myocardial infarction by prolonging the hMSCs' survival time for the treatment [66].

### 3.3. Phosphorylation

Phosphorylation, one of the earliest known PTMs, plays an extensive role in mediating protein activation or deactivation, and is extremely essential for nearly every aspect of cell life. Protein phosphorylation was first identified by Phoebus Levene in 1906, and phosphorylation as a regulatory physiological mechanism was discovered in 1955. Researchers at the time found that converting phosphorylase B to phosphorylase A required phosphate-containing enzymes to interact with ATP. Phosphorylation or dephosphorylation can be reversibly catalyzed by protein kinases or phosphatases, respectively [67, 68]. Unlike the previous modified binding sites, phosphorylation transfers the phosphorylated group to the protein residues of the serine (Ser), threonine (Thr), and tyrosine (Tyr) in the targeted protein, so the phosphorylated protein is negatively charged [69]. Proteins in mitochondria undergo phosphorylation by the catalysis of related enzymes, which significantly affects the occurrence of CVDs [70].

#### 3.3.1. Mitochondrion-Associated Phosphorylation in Myocardial Infarction and I/R Injury

Normal mitochondria produce ATP molecules by oxidative phosphorylation. However, mitochondrial dysfunction produces harmful effects on oxidative phosphorylation and facilitates the generation and accumulation of ROS, thus exacerbating myocardial infarction [71]. Metformin, a drug for the treatment of type 2 diabetes, can alleviate myocardial infarction and improve the survival rate of patients. Evidence revealed that metformin significantly increased phosphorylation of Akt (also known as PKB), thereby inhibiting the opening of mPTP, and it activated the downstream kinase of the reperfusion-induced survival kinase (RISK), thereby alleviating myocardial infarction [72, 73]. Phosphorylation of the mitochondrial complex IV (C_IV_) subunit is essential for maintaining the activity of C_IV_ in myocardial mitochondria. In response to cardiac I/R, protein kinase A-dependent phosphorylation of the IVI1 and VB subunits of C_IV_ were elevated, resulting in a decrease in C_IV_ activity and an increase in ROS production [74, 75]. The signal transducer and activator of transcription 3 (STAT3) plays a key role in regulating mitochondrial metabolism. STAT3 can interact with various mitochondrial proteins and genomes to promote mitochondrial respiration once STAT3 translocated into mitochondria [76]. It has been shown that STAT3 phosphorylation improved mitochondrial function by affecting the mitochondrial complex I (C_I_) in the mitochondrial electron transport chain, preventing the opening of mPTP in the outer membrane, and in turn reducing the myocardial infarction area [77–79]. In addition, phosphorylation of proteins in mitochondria is also involved in cell death. For instance, phosphorylation of a voltage-dependent anion channel (VDAC) protein in the OMM can induce apoptosis that affects the cardiovascular heathy condition [80]. To sum up, mitochondrial phosphorylation elicits a pivotal role in myocardial damage by affecting mitochondrial respiration and quality control.

#### 3.3.2. Mitochondrion-Associated Phosphorylation in Heart Failure

In failing hearts, changes in mitochondrial shape and cristae structure can lead to a reduction in the capacity for energy production [81, 82]. Research by Dey et al. established a nonischemic heart failure model using guinea pigs to mimic human failure. They found that the increase of mitochondrial ROS in heart failure blocked the normal signalling connection between the cytoplasm and the nucleus [83]. Besides, other researchers revealed that the mitochondrial respiratory function of mitochondrial C_I_ and C_II_, as well as the ability of oxidative phosphorylation, were repaired in mice with heart failure following a mild linoleic acid feeding [84]. In addition to a decrease in ATP productivity, another characteristic of heart failure is the accumulation of mitochondrial debris. Evidence suggests that Drp1 phosphorylation facilitates the mitochondrial fission process by promoting its recruitment at OMM in chronic heart failure [85].

### 3.4. Acetylation

Acetylation is one of the major PTMs in cell biology. Basically, acetylation occurs with the transfer of acetyl groups from acetyl coenzyme A (acetyl CoA) to lysine residues of the target protein by acetyltransferase (HAT), causing a conformational change because of the neutralization of their positive charge. Histone acetylation and deacetylation mediated by histone HAT and histone deacetylase (HDAC) are dynamic processes and are directly involved in the regulation of gene transcription. Acetylation can also occur in nonhistone proteins, such as p53, the first acetylated nonhistone protein discovered in 1997 [86]. There are 18 types of HDACs in eukaryotes, which can be divided into four classes, including I, IIa, IIb, and III. Sirtuins (SIRT) are deacetylases belonging to class III HDACs [87]. At present, there are seven subtypes in mammals, namely, SIRT1-SIRT7. Although they are NAD^+^ dependent, they play different roles depending on their distributions in the cell. SIRT3 and SIRT5 are only found in mitochondria, SIRT6 and SIRT7 are only found in the nucleus, while SIRT1 and SIRT2 are found in both the cytoplasm and the nucleus [88]. Importantly, studies have shown that more than half of the proteins in mitochondria have acetylation sites and are closely related to energy metabolism [89–92]. Therefore, acetylation and deacetylation have a high regulatory effect on mitochondrial function, and further affect the occurrence of CVDs.

#### 3.4.1. Mitochondrion-Associated Acetylation in Heart Failure

Lysine acetylation is involved in the regulation of various enzymes related to mitochondrial energy metabolism, in particular, malate dehydrogenase (MDH) and isocitrate dehydrogenase (IDH). Once they are significantly acetylated, however, the expression of SIRT3 and NAD^+^ is significantly decreased [93]. In addition, it is well known that CypD is a sensor for the opening of mPTP channels on the OMM, and CypD activity has a positive correlation with acetylation of mitochondrial protein [94]. A study showed that the activity of CypD was reduced by SIRT3 deacetylation, finally inhibiting the opening of the mPTP channel [95]. Increasing SIRT3 expression in failing hearts can improve cardiac function. Metformin intake significantly increased SIRT3 expression accompanied with reduced PGC-1 acetylation levels, leading to an attenuation of damaged membrane potential and improvement in mitochondrial respiratory function, thereby improving heart function in mice with myocardial infarction-induced heart failure [96]. Therefore, SIRT3 elicits a significant effect on sustaining normal cardiac function.

#### 3.4.2. Mitochondrion-Associated Acetylation in Myocardial I/R Injury

SIRT3 is one of the main pathways of deacetylation and I/R regulation. Studies have shown that the absence of one or two SIRT3 alleles (SIRT3^-/+^ or SIRT3^−/−^) in the heart increases susceptibility to I/R injury. After I/R intervention, myocardial cell injury and infarction area increased, along with decreased cardiac recovery [97, 98]. Zhao et al. investigated the effect of HDAC on cardiac I/R injury by establishing models of early and delayed cardiac pharmacologic preconditioning, respectively. The results revealed that HDAC inhibition protected the heart against I/R injury in both pharmacologic pretreatments [99]. Their follow-up experiments further proved that NF-*κ*B, Akt, and MKK3 are important mediators of HDAC-associated cardiac protection in the delayed preconditioning model [100, 101]. Chang et al. found that *trans*-sodium crocetinate (TSC) reduced cardiac I/R injury by augmenting SIRT3 activity and reducing the phosphorylation and acetylation of FOXO3a protein. The protective effect of SIRT3 can be eliminated by knocking out SIRT3 [102]. In addition, SIRT1 was also found to be involved in cardiac I/R injury. Evidence has shown that the treatment of thymoquinone (TQ) gradually restored left ventricular function by increasing the expression of SIRT1 and the acetylation level of p53 during the construction of myocardial I/R models in rats and suckling mice [103].

#### 3.4.3. Mitochondrion-Associated Acetylation in Cardiac Hypertrophy

Overexpression of SIRT1 can aggravate cardiac hypertrophy, and when decompensated, can eventually induce heart failure. It was found that the activation or upregulation of SIRT1 induced by phenylephrine was inhibited by downregulating or inhibiting AMPK expression, thus alleviating cardiac hypertrophy [104]. Akt is one of the crucial molecules regulating cardiac hypertrophy. The study by Sundaresan et al. indicated that acetylation of Akt and PDK1 blocked their binding to PIP3. The combination of Akt, PDK1, and PIP3 was intensified and activated via deacetylation of Akt by SIRT3, causing cardiac hypertrophy [105]. On the contrary, SIRT3 has the ability of resisting cardiac hypertrophy. Evidence showed that SIRT3 expression was increased in the early stages of cardiac hypertrophy, but it decreased gradually as the disease progressed [106]. Moreover, overexpression of SIRT3 was found to inhibit cardiac hypertrophy, and conversely, knocking out SIRT3 worsened cardiac hypertrophy [107]. Moreover, SIRT6 was reported to reduce the development of cardiac hypertrophy by targeting c-Jun signalling [108]. Since the SIRT family has multiple downstream molecules, the regulation of SIRT on cardiac hypertrophy may vary with different influencing factors.

### 3.5. Succinylation

Succinylation is a new reversible PTM proposed by Zhang et al. in 2011 [109]. It is a natural modification, conservative in evolution. Succinylation occurs with the transfer of the succinyl group to the lysine residue of the receptor protein under the action of succinyl transferase. Succinyl coenzyme A and succinate are known as succinyl donors; however, the enzymes involved in the transfer are not clear. Under physiological pH (7.4), the charge of succinylation of lysine residues is changed from +1 to -1. Lysine succinylation triggers more substantial changes to the structure and chemical properties of a substrate protein compared to other lysine modifications as it formed a mass shift of 100.0186 Da at the Lys residue [109]. It has been found that succinylation is more likely to occur in prokaryotes than in eukaryotes, and in eukaryotes, mitochondria are the organelles with the most succinylation [110]. Importantly, SIRT5, as a mitochondrial deacetylase, also shows the activity of deacetylase, which separates the substrate protein from the succinyl group [111, 112]. Many energy metabolic pathways are closely related to SIRT5-mediated succinylation, such as ATP synthesis and TCA [113]. In SIRT5 overexpressed cells, the levels of mitophagic receptor BCL2 interacting protein 3 (BNIP3) and autophagy marker MAPLC3B decreased, while in contrast, knocking down or inhibiting SIRT5 in cells may affect mitochondrial quality control by accelerating mitophagy [114]. With the analysis of succinylation in recognition sites, evidence has shown that succinylation plays an important role in vascular diseases by regulating various metabolic pathways, although the specific pathway remains to be explored [115, 116].

#### 3.5.1. Mitochondrion-Associated Succinylation in Myocardial I/R Injury

Studies have shown that SIRT5-mediated succinylation plays a protective role in preventing myocardial I/R injury. By comparing different metabonomic methods, succinic acid accumulation has been considered as a common metabolic phenomenon in ischemia tissues due to the effect of succinate dehydrogenase (SDH). However, during reperfusion, the previously existing succinic acid can be oxidized to produce a large amount of ROS, which aggravates myocardial cell damage [117]. When blood flow was restored, injection of dimethyl malonate, a competitive SDH inhibitor, resulted in a significant reduction in myocardial infarct size [117]. Moreover, SIRT5 knockdown in mitochondria of cardiomyocytes increased lysine succinylation and cardiac I/R injury. Succinylated residues on SDH subunit A are the recognition sites of SIRT5. In a word, their study demonstrated that SIRT5 alleviates heart I/R injury by regulating succinylation modification, whereas deletion of SIRT5 promotes mitochondrial death and cardiac anomalies through the accumulation of mitochondrial ROS, which can be alleviated by SDH inhibition [118].

#### 3.5.2. Mitochondrion-Associated Succinylation in Atrial Fibrillation (AF)

AF has a high mortality and incidence rate. The abnormal energy metabolism of cardiomyocytes not only promotes the risk of AF but also increases the probability of heart failure [119]. Previously, research revealed that in SIRT5-deficient hearts, the occurrence of succinylation leads to a large amount of ROS production [117]. However, the increase in ROS can be detrimental to the heart and can accelerate the development of AF [120]. Recently, it has been found that the succinylation levels involved in energy metabolism were significantly altered in AF patients, suggesting a possible correlation between them [121]. Furthermore, changes in succinic acid expression also affect atrial dysfunction and cardiogenic stroke [122]. However, the mechanism of succinylation in AF is still unclear.

#### 3.5.3. Mitochondrion-Associated Succinylation in Cardiac Hypertrophy

ECHA, a subunit of mitochondrial functional proteins required for oxidation of long-chain fatty acids, contains abundant sites for succinylation and can be activated by SIRT5 at Lys351 [115]. SIRT5 knockout decreased the ECHA activity, accompanied with a decrease in fatty acid oxidation, and thus inducing fat accumulation in the heart, contributing to the progression of cardiac hypertrophy [115]. Recently, Hershberger et al. investigated the relationship between SIRT5 and stress overload cardiomyopathy caused by converse aortic treatment (TAC). The results showed that after TAC surgery to SIRT5 knockout mice, cardiac fatty acid metabolism and TCA circulation were impaired, resulting in cardiac hypertrophy [123]. However, because of current limited research, the role of the specific pathway of protein succinylation modification in cardiac hypertrophy needs to be further explored in the future.

### 3.6. Potential Role of Mitochondrion-Related Histone Lactylation in CVDs

Lactic acid is widely known as a metabolite by-product of glucose metabolism. Even under aerobic conditions, glucose can be incompletely oxidized, resulting in the formation of lactate, through a process known as the Warburg effect [124]. In 2019, Zhang et al. identified a novel PTM, lactylation modification, by using high-performance liquid chromatography- (HPLC-) tandem mass spectrometry (MS/MS), immunoblotting analysis, and isotopic localization [125]. The incomplete oxidation product lactic acid of glucose is further converted to lactic acid coenzyme A which is then transferred to histone lysine residues in the presence of acetyltransferase P300 [125]. Recently, a previously unexplored feedback mechanism was discovered that may regulate glycolytic flux under hyperglycaemic or Warburg-like conditions [126]. It has also been reported that histone lactylation plays an essential role in the phenotypic transformation of macrophages [127].

Inflammation is one of the causes and mechanisms that induce cardiac disorders. In the clearance process of inflammatory infiltration, macrophages express repair genes and reduce inflammatory genes to protect host tissues from impairment. Recently, the study of modulating macrophages upon inflammatory response has become more important, and it has involved multiple inflammatory diseases, such as myocarditis [127, 128], atherosclerosis [129], obesity [130, 131], cancer [132], and colitis [133]. In vivo, macrophages can engulf foreign invasion, abnormal microorganisms, or cellular debris to maintain the normal homeostasis of our body system. Basically, there are two phenotypes of macrophages: the M1 macrophage is mainly implicated in proinflammatory responses, while the M2 macrophage is an anti-inflammatory type. Evidence has shown that inflammatory macrophages undergo aerobic glycolysis to generate lactic acid following toll-like receptor stimulation, and then the lactic acids bind to lysine residues in the histone tails, referred to as histone lactylation, which participates in the transformation process of macrophages from M1 to M2 to restore normal cellular functions [134]. In the pathogenesis of pulmonary fibrosis, lactic acid induced histone lactylation in the promoter of the prefibrotic gene in macrophages, which is mediated by P300 [135]. In addition to binding to histones, lactylation can also occur on the sites of nonhistones. Gao et al. found that lactylated proteins in *Botrytis cinerea* are mainly distributed in the nucleus, mitochondria, and cytoplasm, and are correlated with their pathogenicity through protein-protein interactions [136].

### 3.7. Potential Role of Mitochondrion-Related Crotonylation in CVDs

Another new PTM, lysine crotonylation, was discovered by Tan et al. in 2011. This modification mainly functions in the nucleus and can be detected at multiple histone sites [137]. Lysine crotonylation is enzymatically regulated by the dynamic balance between crotonyl transferases (writer) and decrotonylases (eraser). The crotonyl transferases catalyze the formation, whereas the decrotonylases catalyze the removal of the covalent modification of the crotonylation [138]. Some studies have found that several deacetylases including HDAC1, HDAC2, and HDAC3 also have the activity of decrotonylases, which are regarded as major executors of histone decrotonylation [139–141]. Several proteins that function as crotonyl transferases have also been identified, such as P300, MOF, and CBP [142]. Andrews et al. found that the Taf14 YEATS domain can act as a reader of histone crotonylation [143]. In particular, YEATS domains recognize histone crotonylation by a unique mechanism of aromatic-*π* stacking, linking crotonylation to transcription, nucleosome remodeling, and other important cellular functions [144]. The histone crotonylation induced by crotonic acid can activate Zscan4 to maintain telomeres and promote CiPSC generation, indicating that the crotonylation facilitates telomere maintenance and enhances chemically induced reprogramming to pluripotency [145]. Nevertheless, the current studies about crotonylation mainly focus on its effects on the nucleus and on protein coding; however, the precise role of crotonylation in CVDs has not been well demonstrated, which may be worth exploring in the future.

## 4. Clinical Perspective and Application of PTMs in CVDs and Other Diseases

With rapid progress in proteomics and mass spectrometry-based technology, a large number of PTMs have been found in human gene products by means of protein profiling techniques [146]. Until 2015, the UniProt database has recorded 469 PTMs including 326 PTMs in eukaryotes and more than 100 different PTMs in *Homo sapiens* [147], suggesting a potential clinical research direction for human diseases. It has been proven that PTMs are closely related to the occurrence of human diseases, such as cancer, diabetes, and CVDs [148–150]. To this end, it is critical for researchers to carry out biomarker discovery through characterization and quantitation of PTMs. PTMs thus exhibit an applicable role in the prediction of CVDs or other diseases by detecting the expression level of circulating PTM proteins or their specific molecular regulators, and may further provide therapeutic approaches by altering the degree of specific protein modifications for disease treatment.

## 5. Summary and Conclusions

In recent years, with growing numbers of in-depth studies on PTMs, more types of PTMs have gradually been discovered. To make a better understanding of their roles in CVDs, we summarized the current research progress of several major PTMs that affect CVDs by regulating specific mitochondrial proteins which are closely implicated in mitochondrial quality control (see Table 1). The heart is an important organ which requires enough energy supplies provided by mitochondria in cardiomyocytes. Abnormal mitochondrial quality control may contribute to the development of different types of CVDs. Since most PTMs are reversible, it enables us to control the direction of each reaction by regulating different enzymes for the disease intervention based on their particular pathogenesis. Interestingly, lactylation and crotonylation as two novel PTMs that were discovered recently [125, 137], are closely associated with mitochondrial metabolism, although the precise regulating mechanism and their role participating in CVDs have not been explored yet. In line with this notion, different types of PTMs are not completely independent during the regulation process in CVDs or other disorders. They have complex networks of interactions, especially by modulating several essential mitochondrion-related proteins or enzymes. For instance, the PINK-mediated Parkin pathway exhibits a critical role in regulating not only the mitophagy but also the PTM progress, such as SUMOylation and ubiquitination. Parkin maintains the normal function of mitochondria by inhibiting the opening of mPTP by catalyzing the ubiquitination of CypD in the necrotic cascade, while phosphorylation of PINK1 recruits Parkin to depolarize mitochondria and increase the mitophagy process. The ubiquitin protein itself can also be phosphorylated by PINK, along with the phosphorylation of Parkin at serine-65 (Ser65). This process mediates Parkin activation and recruitment as well as E3 Ub ligase activity [151]. On the other hand, PTMs can also affect proteins that are associated with mitochondrial fusion and fission such as OPA1 (see Figure 3). Acetylation and succinylation normally occur at the lysine residues of the target protein and are closely associated with SIRT activity and energy metabolism. However, although these mitochondrial proteins are mostly involved in the regulation of mitochondrial quality control including mitochondrial fission, fission, mitophagy, and biogenesis, we cannot exclude other proteins modified by different PTMs (some are not described in this review) which may directly or indirectly affect the mitochondrial quality control. Nevertheless, the investigation on the interaction network of PTMs in CVDs by modulating mitochondrial quality control has a promising future en route to exploring novel therapeutic targets.

## Figures and Tables

**Figure 1:** The process of protein SUMOylation. First, the inactive SUMO protein is activated by the action of SENPs. By consuming 1 molecule of ATP, a SUMO protein binds to the E1 activating enzyme. The E2 conjugating enzyme replaces E1 to bind to the SUMO protein. Then, E2 presents the SUMO protein to the E3 ligase, which specifically recognizes the target protein and makes SUMO bind to the Lys residue on the target protein to achieve the goal of protein structural and functional changes. SENPs are also required for the deSUMOylation process.

**Figure 2:** The process of protein ubiquitination. First, the inactive ubiquitin (Ub) molecule is activated under the catalysis of DUBs. Under the action of 1 molecule of ATP, Ub binds to an E1 activating enzyme; then, the E2 conjugating enzyme replaces E1 and connects to Ub. Next, E2 presents Ub to the E3 ligase, and the E3 ligase binds specifically to the target protein. The above steps are repeated until the target protein binds more than 4 Ub molecules to form a Ub chain. Then, the 26S proteasome recognizes the Ub chain and places the target protein in its own barrel. Finally, the target protein is degraded into small fragments by ATP consumption, and the Ub molecule is restored for release.

**Figure 3:** The role of posttranscriptional modification of mitochondrial proteins in mitochondrial quality control. The quality control of mitochondria mainly includes fusion, fission, mitophagy, and biogenesis. Ubiquitination of the mitochondrial protein OMA1 promotes the fusion of healthy mitochondria. The ubiquitination of mitochondrial protein AKAP121 and the phosphorylation of Drp1 are conducive to the fission of normal mitochondria. Phosphorylation of mitochondrial protein PINK1 and SUMOylation of Drp1 induces mitophagy in unhealthy mitochondria.

**Table 1:** The relationships between PTMs of mitochondrial proteins and cardiovascaular diseases.

Mitochondrial proteins	PTMs	Upstream regulators	Impacts on mitochondrial quality control	Mechanism	Cardiovascular diseases	Roles in cardiovascular diseases	References
Drp1	SUMOylation	SUMO1	Positive	Induce autophagy	I/R injury	Weaken myocardial I/R intervention	[43]
Drp1	SUMOylation	SENP5	Positive	Inhibit the activation of apoptosis factor	Heart failure	Relieve heart failure	[47]
CypD	Ubiquitination	Parkin	Positive	Inhibit the opening of mPTP	I/R injury	Alleviate heart I/R injury	[56]
OMA1	Ubiquitination	GSK3	Positive	Increase OPA1 expression	Heart failure	Relieve heart failure	[66]
AKAP121	Ubiquitination	ACSL1	Negative	Increase mitochondrial division	Cardiomyopathy	Promote the formation of lipotoxic cardiomyopathy	[64]
Cytochrome C oxidase	Phosphorylation	PKA	Negative	Increase ROS production	I/R injury	Increase myocardial I/R injury	[74, 75]
STAT3	Phosphorylation	Unclear	Positive	Improve the respiration of C_I_, inhibit the opening of MPTP		Relieve myocardial I/R injury	[77–79]
VDAL	Phosphorylation	HK2	Negative	Promote apoptosis		Aggravate heart I/R injury	[80]
Akt	Phosphorylation	PI3K	Positive	Inhibit the opening of mPTP	Myocardial infarction	Alleviate myocardial infarction	[72, 73]
PINK1	Phosphorylation	AMPK*α*2	Positive	Induce autophagy	Heart failure	Relieve heart failure	[65]
Drp1	Phosphorylation	PKA	Negative	Increase mitochondrial division		Aggravate heart failure	[85]
GSK3*β*	Acetylation	SIRT3	Positive	Reduce cardiac fibrosis	Heart failure	Relieve heart failure	[93]
CypD	Acetylation	SIRT3	Negative	Induce the opening of mPTP	Heart failure	Aggravate heart failure	[95]
PGC-1*α*	Acetylation	SIRT3	Negative	Destroy mitochondrial membrane potential		Aggravate heart failure	[96]
FOXO3a	Acetylation	SIRT3	Negative	Oxidative damage to mitochondria	I/R injury	Aggravate myocardial I/R injury	[102]
P53	Acetylation	SIRT1	Negative	Promote ROS production		Accelerate myocardial I/R injury	[103]
Akt/PDK1	Acetylation	SIRT1	Positive	Prevent Akt/PDK1 from combining with PIP3	Myocardial hypertrophy	Reduce myocardial hypertrophy	[105]
SDH	Succinylation	SIRT5	Positive	Decrease ROS production	Atrial fibrillation	Relieve myocardial I/R injury	[118]
Unknown	Succinylation	Unknown	Negative	Increase ROS production		Accelerate myocardial I/R injury	[120]
ECHA	Succinylation	SIRT5	Unknown	Accelerate oxidation of fatty acids	Myocardial hypertrophy	Weaken myocardial hypertrophy	[115]
